RETRACTED

# Ruptured Isolated Common Iliac Artery Aneurysm Masquerading as Renal Colic

**DOI:** 10.7759/cureus.19752

**Published:** 2021-11-19

**Authors:** Mohanned F Alfahhad, Halimah A Qasem, Nermeen N Alrajhi, Luay T Khayat, Meaad K Alsulami, Salem A Al Marri, Hassan M Alshuqaybi, Saad R Aldhafyan, Fahad M Al Jabir, Naif A Albaqami, Atheer M Alyami, Abrar M Alamrani, Dina N Abusabir, Adnan N Alkhaldi, Faisal Al-Hawaj

**Affiliations:** 1 College of Medicine, King Abdulaziz University, Jeddah, SAU; 2 College of Medicine, Jazan University, Jazan, SAU; 3 College of Medicine, King Saud Bin Abdulaziz University For Health Sciences, Jeddah, SAU; 4 College of Medicine, King Faisal University, Al-Ahsa, SAU; 5 College of Medicine, King Saud Bin Abdulaziz University For Health Sciences, Riyadh, SAU; 6 College of Medicine, Vision Colleges, Riyadh, SAU; 7 College of Medicine, University of Tabuk, Tabuk, SAU; 8 College of Medicine, King Saud University, Riyadh, SAU; 9 College of Medicine, Imam Abdulrahman Bin Faisal University, Dammam, SAU

**Keywords:** case report, laparotomy, common iliac artery, hematoma, aneurysm, flank pain

## Abstract

Urinary stone disease is a common problem globally. Ureteric colic typically presents with flank pain and hematuria. However, several conditions may give a similar clinical picture. Hence, imaging studies are essential to make the diagnosis of urinary stone disease and evaluate for possible complications. We present the case of a 64-year-old man who presented with severe left flank pain radiating to the groin for two days. In his first visit to the emergency department, he was prescribed conservative treatment, but it failed to give any clinical improvement. The patient does not have a previous history of urinary stone disease. He had a long-standing history of hypertension, diabetes mellitus, dyslipidemia, and coronary artery disease. Further, he had a 30 pack-years history of smoking. Upon examination, the abdomen was soft and lax with generalized tenderness. Subsequently, a non-contrast computed tomography scan for the kidneys, ureters, and bladder was performed, which demonstrated a large high attenuation fluid seen in the left side of the retroperitoneum. The scan was then repeated after the administration of intravenous contrast and showed an aneurysmal dilatation of the left common iliac artery with surrounding hematoma. The patient was taken for an emergency laparotomy for evacuation of the hematoma and graft repair of the aneurysm. The patient tolerated the operation without complications. The present case highlights the importance of considering the wide differential diagnoses of flank pain in emergency settings. Physicians should keep a high index of suspicion for aneurysmal disease when they encounter patients with risk factors for arterial wall degeneration.

RETRACTED

## Introduction

Urinary stone disease is a common problem worldwide. It affects up to 20% of men during their lifetime [1]. Ureteric stones have the classic presentation of flank pain and hematuria. Diagnostic studies are needed to accurately diagnose the stone disease and to evaluate for its possible complications. The first-line imaging study is a non-contrast computed tomography scan of the kidneys, ureters, and bladder using a low radiation dose [2]. Numerous conditions may give a similar clinical picture to ureteric stones [3]. Such conditions commonly include non-stone genitourinary causes (e.g., renal tumors), gynecologic conditions (e.g., ruptured ovarian cyst), and gastrointestinal diseases (e.g., acute diverticulitis). Furthermore, hepatobiliary, musculoskeletal conditions should be considered. Vascular diseases causes must always be considered in patients with renal colic because these conditions can be life-threatening emergencies. Serious vascular conditions like abdominal aortic aneurysm and renal infarction may present with acute flank pain and hematuria. Here, we report the case of an elderly man who had a ruptured isolated common iliac artery aneurysm masquerading as renal colic.

## Case presentation

We present the case of a 64-year-old man who presented to the emergency department because of severe left flank pain radiating to the groin for two days duration. The pain was burning in nature and had been increasing in severity. He rated the pain as 9 on the 10-point severity scale. The pain was constant and was not related to posture, meal intake, or urination. The patient visited the emergency department earlier that day and he was discharged with conservative measures and was given an appointment with the urology team. However, the pain progressed in severity and it became intolerable. Further, the prescribed analgesics failed to provide any clinical improvement. There was no history of change in the urine color or fever. The patient did not have any history of urinary stone disease. He had a long-standing history of diabetes mellitus, hypertension, and dyslipidemia. He also had a history of coronary artery disease for which he underwent percutaneous coronary intervention. The patient had poor control of these conditions and his compliance to medications was poor. He had not undergone any previous surgeries. He was not known to have any drug or food allergies. He was a retired teacher. The patient had a 30 pack-years history of smoking. He had never consumed alcohol. His family history was non-contributory.

RETRACTED

Upon examination, the patient appeared in pain. His vital signs revealed tachycardia (128 bpm), tachypnea (18 bpm), normal temperature (37.1℃), and maintained blood pressure (110/75 mmHg). The abdomen was soft and lax with generalized tenderness. The cardiorespiratory examination was unremarkable. The urine dipstick indicated the presence of red blood cells with negative leukocyte esterase and nitrites. Initial laboratory markers showed hemoglobin of 14.1 g/dL, leukocytes count of 8,000/μL, and platelets count of 380,000/μL. Other biochemical parameters, including liver enzymes, urea, and electrolytes, were within the normal limits (Table 1).

**Table 1:** Summary of the results of laboratory findings

Laboratory Investigation	Unit	Result	Reference Range
Hemoglobin	g/dL	14.1	13.0–18.0
Leukocytes	1000/mL	8.0	4.0–11.0
Platelet	1000/mL	380	140–450
C-Reactive Protein	mg/dL	8.5	0.3–10.0
Erythrocyte Sedimentation Rate	mm/hr.	14.5	0–20
Albumin	g/dL	4.5	3.4–5.0
Total Bilirubin	mg/dL	0.8	0.2–1.2
Alanine Transferase	U/L	22	14–63
Aspartate Transferase	U/L	21	15–37
Gamma-glutamyltransferase	U/L	17	15–85
Alkaline Phosphatase	U/L	50	46–116
Creatinine	mg/dL	0.9	0.7–1.3
Blood Urea Nitrogen	mg/dL	12	7–18
Serum Sodium	mEq/L	135	136–145
Serum Potassium	mEq/L	3.9	3.5–5.1
Serum Chloride	mEq/L	104	98–107

The patient was seen by the Urology Team for suspected renal colic. Non-contrast computed tomography scan for the kidneys, ureters, and bladder was performed. The scan demonstrated a large high attenuation fluid seen in the left side of the retroperitoneum suggestive of a hematoma (Figure 1). Subsequently, the scan was repeated in the arterial phase after the administration of intravenous contrast. It showed an aneurysmal dilatation of the left common iliac artery with surrounding hematoma (Figure 2). The contralateral common iliac artery and the abdominal aorta were normal. The patient was taken for an emergency laparotomy. The hematoma was evacuated and a Dacron graft of the affected artery was successfully inserted. The patient had a successful recovery. The patient was discharged on the fourth postoperative day. After three months of follow-up, the patient had no active complaints.

**Figure 1:** Coronal image of a non-contrast CT abdomen demonstrating a localized large high attenuation fluid (arrow) seen in the left side of the retroperitoneum suggestive of a hematoma

**Figure 2:** Axial contrast-enhanced CT image demonstrating aneurysmal dilatation of the left common iliac artery (arrow) with surrounding hematoma

## Discussion

We presented the case of a ruptured isolated left common iliac artery aneurysm with a clinical picture suggestive of ureteric colic. Isolated iliac artery aneurysm is rare and accounts for less than 1% of all cases of aneurysmal disease [4]. However, concomitant aortic and iliac aneurysms are not uncommon and have an estimated prevalence of 1% in adults [5].

RETRACTED

The risk factors for developing an iliac artery aneurysms are similar factors for other large vessel aneurysms. In the present case, advanced age, male sex, hypertension, coronary artery disease, and smoking were predisposing factors for the formation and expansion of the iliac artery aneurysm. In a retrospective study by Patel et al. [6] on cases of common iliac artery aneurysms, they found that >90% of patients were men, 80% had hypertension, and 60% were smokers. Regarding the clinical manifestation of common iliac artery aneurysms, previous studies suggest that nearly half of patients are asymptomatic and have the aneurysm detected incidentally on imaging, and one-third of cases present with rupture [7]. Larger aneurysms are more likely to be symptomatic. The symptoms of aneurysms can be related to its compression of adjacent structures, thrombosis, thromboembolism, and rupture.

In more than 70% of cases of iliac artery aneurysm, the patient is found to have a pulsatile mass on abdominal examination [7]. However, as in our case, the absence of the pulsatile mass does not rule out the diagnosis of the iliac aneurysm. Considering the non-specific presentation of iliac aneurysms, imaging studies are vital to establishing the diagnosis. Ultrasound examination of the abdomen and pelvis can demonstrate the aneurysmal disease, but it is often limited because of the overlying bowel gas that obscures the findings [8]. In our case, the diagnosis was reached by computed tomography scan that was performed for ruling out urinary stone disease.

Early diagnosis of iliac artery aneurysm is vital to reduce the mortality risk. Ruptured and symptomatic aneurysms require emergency repair while careful surveillance may be done for small asymptomatic aneurysms. The presence of a co-existing abdominal aortic aneurysm is taken into consideration for planning the management of the iliac artery aneurysm. Both open and endovascular approaches have been described in the management of iliac artery aneurysms [4]. In the present case, an open approach was performed because of the surgeon’s experience and preference.

## Conclusions

The present case highlights the importance of considering the wide differential diagnoses of flank pain in emergency settings. Physicians should keep a high index of suspicion for aneurysmal disease when they encounter patients with risk factors for arterial wall degeneration, including advanced age, male gender, hypertension, and smoking. A computed tomography scan can diagnosis an aneurysmal disease accurately. Early diagnosis is vital since prompt repair of the ruptured aneurysm is of paramount importance to save the patient life.
